This article has been retracted.

# microRNA-18a from M2 Macrophages Inhibits TGFBR3 to Promote Nasopharyngeal Carcinoma Progression and Tumor Growth via TGF-β Signaling Pathway

**DOI:** 10.1186/s11671-020-03416-8

**Published:** 2020-10-02

**Authors:** Ya Peng, Xiangsheng Li, Huowang Liu, Xiaowen Deng, Chang She, Chenxi Liu, Xinxing Wang, An Liu

**Affiliations:** 1 Department of Otolaryngology Head and Neck Surgery, Affiliated Changsha Hospital of Hunan Normal University, The Fourth Hospital of Changsha, Changsha, Hunan 410006 People’s Republic of China; 2 Department of Otolaryngology Head and Neck Surgery, Third Xiangya Hospital, Central South University, 138th Tongzipo Road, Yuelu District, Changsha, Hunan 410013 People’s Republic of China; 3 5th Department of Cardiology, Hunan Provincial People’s Hospital, The First Affiliated Hospital of Hunan Normal University, Changsha, Hunan 410005 People’s Republic of China; 4 Third Xiangya Hospital, Central South University, 138th Tongzipo Road, Yuelu District, Changsha, Hunan 410013 People’s Republic of China

**Keywords:** Nasopharyngeal carcinoma, M2 macrophages, MicroRNA-18a, Transforming growth factor-beta III receptor, Transforming growth factor signaling pathway, Viability, Apoptosis, Migration, Invasion

## Abstract

**Objectives:**

Nasopharyngeal carcinoma (NPC) is a type of nasopharyngeal disease with high metastasis and invasion properties. Tumor-associated alternative activated (M2) macrophages are evidenced to connect with NPC. Based on this, this study purposes to explore the mechanism and participation of microRNA-18a (miR-18a) from M2 macrophages in NPC.

**Methods:**

Peripheral blood mononuclear cells were differentiated to macrophages and macrophages were polarized to M2 type by interleukin-4. SUNE-1 and CNE2 cells were transfected with restored or depleted miR-18a or transforming growth factor-beta III receptor (TGFBR3) to explore their roles in NPC progression with the involvement of the TGF-β signaling pathway. Next, SUNE-1 and CNE2 cells were co-cultured with M2 macrophages that had been treated with restored or depleted miR-18a or TGFBR3 to comprehend their combined roles in NPC with the involvement of the TGF-β signaling pathway.

**Results:**

MiR-18a was highly expressed and TGFBR3 was lowly expressed in NPC cells. MiR-18a restoration, TGFBR3 knockdown or co-culture with miR-18a mimics, or si-TGFBR3-transfected M2 macrophages promoted SUNE-1 cell progression, tumor growth in mice, decreased p-Smad1/t-Smad1, and elevated p-Smad3/t-Smad3. miR-18a downregulation, TGFBR3 overexpression, or co-culture with miR-18a inhibitors or OE-TGFBR3-transfected M2 macrophages depressed CNE2 cell progression, tumor growth in mice, increased p-Smad1/t-Smad1, and decreased p-Smad3/t-Smad3.

**Conclusion:**

Our study elucidates that miR-18a from M2 macrophages results in promoted NPC cell progression and tumor growth in nude mice via TGFBR3 repression, along with the Smad1 inactivation and Smad3 activation.

## Introduction

Nasopharyngeal carcinoma (NPC) is an epithelial malignant tumor that is inclined to local infiltration and early distant metastasis [1]. NPC patients often complain sixth nerve palsy and Horner’s syndrome [2]. At present, the applied treatment predominantly consists of radiotherapy, and integrated radiotherapy and chemotherapy [3]. Unfortunately, radiotherapy and chemotherapy are unexpectedly accompanied by complications, and acquired resistance to radiotherapy hampers the outcomes of NPC [3]. Given that the task to delve out potential targeted therapy ranks a priority.

Dysregulated microRNAs (miRNAs) are documented to be involved in NPC tumorigenesis, metastasis, invasion, and resistance to radiotherapy and chemotherapy [1]. As a subfamily of miRNAs, miR-18a is found to facilitate NPC progression through suppressor of morphogenesis in genitalia 1 inhibition and mTOR pathway activation [4]. Besides that, miR-18a is further verified to activate NPC cell proliferation and metastasis via DICER1 regulation [5]. Additionally, NPC cell progression is evidenced to be driven by miR-18a through miRNA biogenesis impairment [6]. Moreover, miR-18a has been documented to function critically in the metastasis of NPC [7]. Alternative activated (M2) macrophages are important components of solid and hematological malignancies and are connected with progression, metastasis, and therapy resistance [8]. M2-polarized tumor-associated macrophages are associated with poor prognosis of NPC [9]. It is intriguingly recorded the differences of M2 macrophages in Epstein-Barr virus-negative and Epstein-Barr virus-positive NPC [10]. There is a study outlining that miR-18a inhibits liver metastasis of colon cancer cells by inducing M1 macrophages [11]. Transforming growth factor-beta III receptor (TGFBR3) is a TGF-β co-receptor that provides the type II TGF-β receptor ligand to stimulate signaling and balance of cell surface, and soluble TGFBR3 is a regulator during cancer progression [12]. Lowly expressed TGFBR3 is reported to induce an immunotolerant tumor microenvironment [13]. Oppositely, transient overexpression of TGFBR3 induces apoptosis in human NPC cells [14]. To our best knowledge, M2 macrophages polarization induced by miR-181a advances M2 macrophage-mediated tumor cell metastasis via Kruppel-like factor 6 and CCAAT/enhancer binding protein α axis [15].

Collectively, though many studies have discovered the independent role of miR-18a, TGFBR3 and M2 macrophages in NPC, the combined interactions among these three factors are still elusive. Considering that this study is launched to decipher the mechanisms and participation of these factors in NPC.

## Materials and Methods

### Ethics Statement

The experiment was approved by the ethics committee of Third Xiangya Hospital, Central South University and met the medical ethics standards. This study was conducted with written consent from all donors. Animal experiments were in compliance with the requirements of the National Laboratory Animal Management and Use regulations.

### Collection of Peripheral Blood Mononuclear Cells

The monocytes were obtained from peripheral blood of healthy donors by adherent method. Peripheral blood specimens were obtained from healthy donors of the Department of Hematology of Third Xiangya Hospital, Central South University. Monocytes-derived macrophages were obtained through plastic adherence of peripheral blood mononuclear cells (PBMCs) previously isolated by density gradient centrifugation (Ficoll-Paque, GE Healthcare) from buffy coat preparations of blood from healthy donors. Then, 2.0 × 10^6^ PBMCs were cultured in Dulbecco’s modified Eagle medium (DMEM) supplemented with 10% human serum (Millipore, Bedford, MA, USA) and penicillin/streptomycin on 12-well plates (NalgeNunc, NY, USA). When PBMCs were adhered to the wall for 2–3 h, the supernatant and suspended PBMCs were removed repeatedly to obtain adherent monocytes.

### Macrophage Polarization

Monocytes were induced to differentiate into macrophages by human macrophage colony-stimulating factor (M-CSF) and polarized into M2 macrophages by interleukin (IL)-4.

### Induction of Macrophages

Monocytes were cultured in 20% fetal bovine serum (FBS)-DMEM and added with M-CSF (100 μg, Peprotech, NJ, USA) to the final concentration of 100 ng/mL. The medium was renewed in half every 3 days and then supplemented with 100 ng/mL M-CSF. Cultivated to the 7–8th day, part of cells were harvested, and macrophage surface markers CD68 [16], CD163 [17], and CD206 [18] were tested by immunofluorescence assay [19] to identify macrophages.

### Polarization of Macrophage

Macrophages were polarized to M2 macrophages by supplementing 20 ng/mL IL-4 (Peprotech) to the differentiation media for another 24 h. A part of the M2 macrophage samples were utilized for flow cytometry detection. The samples were divided into 3 tubes: tube 1 was the same batch of adherent macrophages without IL-4 stimulation; tubes 2 and 3 were the adherent macrophages stimulated by IL-4. The samples were diluted to about 10,000 cells when loading and added with non-specific immunoglobulin G to block the Fc receptor. Then the samples were added with non-specific isotype antibody, PE-labeled CD68 antibody, and PE-labeled CD163 antibody (both from Biolegend, CA, USA). Incubated for 30 min and rinsed with 0.5% bovine serum albumin in phosphate-buffered saline (PBS), the samples were centrifuged and made into cell suspension with 500 μL PBS for detection.

### Reverse Transcription Quantitative Polymerase Chain Reaction

Reverse transcription quantitative polymerase chain reaction (RT-qPCR) was employed to detect miR-18a, CCL22, peroxisome proliferator-activated receptor γ (PPAR-γ), and TGFBR3 mRNA expression in the collected cells.

Total RNA was extracted from cells by Trizol (Invitrogen, Carlsbad, CA, USA) and reversely transcribed into complementary RNA by Mir-X miRNA First Strand Synthesis Kit (Clontech, Mountain View, CA, USA) for miR-18a and the PrimeScriptTM RT Master Mix Kit (Takara, Dalian, China) for CCL22, PPAR-γ, and TGFBR3. U6 and glyceraldehyde-3-phosphate dehydrogenase (GAPDH) were loading controls for miR-18a, CCL22, PPAR-γ, and TGFBR3. SYBR^@^Premix Ex Taq™ II (Perfect Real Time) (Takara) in a LightCycler 480 II system (Roche Diagnostics, Indiana, USA) was utilized in PCR. Data calculation was evaluated by 2^-△△CT^ method. PCR primers were presented in Table 1.

**Table 1:** Primer sequence

Genes	Primer sequence (5′-3′)
CCL22	Forward: ATTACGTCCGTTACCGTCTG
	Reverse: TAGGCTCTTCATTGGCTCAG
PPAR-γ	Forward: GCCTTGCAGTGGGGATGT
	Reverse: CTCGCCTTTGCTTTGGTC
miR-18a	Stem-loop primer: GTCGTATCCAGTGCAGGGTCCGAGGTATTCGCACTGGATACGACCTATCT
	Forward: GTGCTAAGGTGCATCTAGTGCAG
	Reverse: GTGCAGGGTCCGAGGT
TGFBR3	Forward: CAAAGCAGCAGAAGGGTGTGT
	Reverse: GGTGATTAGCTCGATGATGTGTACTT
U6	Forward: ATTGGAACGATACAGAGAAGATT
	Reverse: GGAACGCTTCACGAATTTG
GAPDH	Forward: GACAACAGCCTCAAGATCATCAG
	Reverse: GTGGCAGTGATGGCATGGA

*PPAR*-*γ* peroxisome proliferator-activated receptor γ, *miR*-*18a* microRNA-18a, *TGFBR3* transforming growth factor-beta III receptor, *GAPDH* glyceraldehyde-3-phosphate dehydrogenase

### Western Blot Assay

Western blot assay was applied to the detection of TGFBR3, total (t)-Smad1, phosphorylated (p)-Smad1, t-Smad3, and p-Smad3 protein in the collected cells.

Total protein of cells was extracted and the protein concentration was determined based on the bicinchoninic acid kit. The protein sample was loaded to the wells in sodium dodecyl sulphate polyacrylamide gel electrophoresis and transferred to a polyvinylidene fluoride (PVDF) membrane. The PVDF membrane was blocked with skim milk and incubated with primary antibodies TGFBR3 (1:2000, R&D Systems, Minneapolis, MN, USA), t-Smad1 (1:1000), p-Smad1 (1:1000, Santa Cruz Biotechnology), t-Smad3 (1:1000), p-Smad3 (1:1000), and GAPDH (1:1000, all from Abcam, Cambridge, MA, UK) which was followed by incubation with the horseradish peroxidase-labeled secondary antibody (1:500, Jackson ImmunoResearch Laboratories, PA, USA). Washed 3 times by tris-buffered saline with Tween 20, the membrane was developed by enhanced chemiluminescence. Quantification of signals was completed by the National Institutes of Health ImageJ Imaging. Processing Analysis Software with signaling intensity normalized to GAPDH.

### Cell Culture and Screening

Human NPC cell lines CNE2, TW03, C666-1, and SUNE-1 and normal human nasopharyngeal cell line NP96 (Shanghai Institutes for Biological Sciences, Chinese Academy of Sciences, Shanghai, China) were cultured in Roswell Park Memorial Institute (RPMI)-1640 medium (Gibco, CA, USA) containing FBS (Gibco), 100 μg/mL penicillin and 100 μg/mL streptomycin and passaged upon 80% confluence. RT-qPCR was utilized to detect miR-18a expression. Among those NPC cell lines, CNE2 and SUNE-1 cells showed largest and smallest difference in miR-18a expression from NP96 cells, thus they were selected for miR-18a down-regulation or up-regulation assays.

### Cell Grouping and Treatment

Among all NPC cell lines, SUNE-1 cells with the smallest difference from NP96 cells in miR-18a expression were selected. Guided by specifications of Lipofectamine 2000 (Invitrogen), SUNE-1 cells were transfected with miR-18a mimics, miR-18a mimics negative control (NC), si-TGFBR3, or si-TGFBR3 NC.

Among all NPC cell lines, CNE2 cells with the largest difference from NP96 cells in miR-18a expression were selected and transfected with miR-18a inhibitors, miR-18a inhibitors NC, overexpression (OE)-TGFBR3 or OE-TGFBR3 NC by Lipofectamine 2000 (Invitrogen).

Guided by specifications of Lipofectamine 2000 (Invitrogen), M2 macrophages were transfected with miR-18a mimics, miR-18a mimics NC, si-TGFBR3, si-TGFBR3 NC, miR-18a inhibitors, miR-18a inhibitors NC, OE-TGFBR3, or OE-TGFBR3 NC.

### Co-culture of M2 Macrophages and NPC Cells

Cell co-culture in the Transwell chamber was adopted to explore the effects of miRNA from M2 macrophage on NPC cells. The upper chamber was filled with M2 macrophage with the pore size being 0.4 μm, which only stopped cells of the upper chamber from passing through but not the small molecules secreted by the cells such as vesicles, growth factors, nutrients, etc. The lower chamber was spread with NPC cells.

SUNE-1 and CNE2 were incubated in normal FBS (Gibco). The cells in the logarithmic growth phase were adopted for experiments.

SUNE-1 and CNE2 cells were co-cultured with M2 macrophages in 10% FBS-RPMI-1640 medium (both from Gibco) in a Transwell insert cell culture dish (Coring, Corning, NY, USA) with a pore size of 0.4 μm.

SUNE-1 cells were not co-cultured with M2 macrophages, or co-cultured with M2 macrophages, miR-18a mimics-transfected M2 macrophages, miR-18a mimics NC-transfected M2 macrophages, si-TGFBR3-transfected M2 macrophages, or si-TGFBR3 NC-transfected M2 macrophages.

CNE2 cells were not co-cultured with M2 macrophages, or co-cultured with M2 macrophages, miR-18a inhibitors-transfected M2 macrophages, miR-18a inhibitors NC-transfected M2 macrophages, OE-TGFBR3-transfected M2 macrophages, or OE-TGFBR3 NC-transfected M2 macrophages.

### 3-(4, 5-Dimethylthiazol-2-yl)-2, 5-Diphenyltetrazolium Bromide Assay

Cell viability was tested by 3-(4, 5-dimethylthiazol-2-yl)-2, 5-diphenyltetrazolium Bromide (MTT) assay, which was a colorimetric assay applied to determine the activity of mitochondrial dehydrogenase, which reduced MTT to formazan.

Trypsinized and seeded into 96-well plates at 4 × 10^4^ cells/well, cells were deprived of culture medium on the 0, 12th, 24th, 36th, and 48th h, respectively and supplemented with MTT solution (500 μL, 0.5 g/L). Incubated for 4 h, the supernatant was discarded and cells were incubated with 200 μL dimethyl sulfoxide solution. Optical density (OD, 490 nm) values were measured on a microplate reader (ELX808IU, BioTek, VT, USA). Each group was set up with 6 parallel wells.

### Colony Formation Assay

Colony-forming ability of NPC cells was tested by colony formation assay, which reflected cell population dependence and cell clonal proliferation.

Cultured for 24 h and detached with 0.25% trypsin, 300 cells were seeded in a 35-mm dish with 3 parallel wells in each group. With culture medium renewed every 3 days, the cells were cultured for a week and fixed with 5 mL 4% paraformaldehyde. After that, the cells were stained by crystal violet staining solution and air dried. The dish was inverted on which a transparent film of grids was superimposed, and the number of colonies (more than 50 cells) was counted under a microscope (Olympus, Tokyo, Japan).

### Scratch Test

Cell migration was tested by scratch test. Cells were trypsinized, seeded into 6-well plates with 3 parallel wells for each group, and cultured to 90% confluence. Then, the cells were incubated in the medium with 2% FBS and vertical scratches were drawn by a 100-μL tip. The cells were photographed on the 0 and 24th h under an inverted microscope to measure cell migration distance.

### Transwell Assay

Cell invasion and migration were tested by Transwell assay. The upper chamber of the Transwell chamber was pre-immersed and added with 100 μL Matrigel (Coring) which had diluted by serum-free RPMI 1640 medium at 1:100. The upper and lower chambers were added with 200 μL and 600 μL serum-free RPMI 1640 medium severally. Subsequently, the lower chamber was added with 600 μL RPMI 1640 medium containing 10% FBS while the upper chamber with 200 μL cell suspension (12.5 × 10^4^ cells/mL). Incubated for 40 h, the cells were stained by crystal violet staining solution and wiped with a cotton swab to count the cells passing through the Matrigel under a microscope.

### Flow Cytometry

Cell apoptosis and cell cycle distribution were determined by flow cytometry.

Cell cycle distribution was evaluated by propidium iodide (PI) staining. Cells were seeded into 6-well plates at 4 × 10^5^ cells/well, and cultured to 70–80% confluence. Fixed in pre-cooled 70% ethanol overnight, the cells were centrifuged (the supernatant was discarded), added with RNAase (1 g/L, 200 μL) and Triton X-100 (2 μL), and stained by PI staining solution for 30 min. After that, cell cycle distribution was detected by a flow cytometer (BD Bioscience, NJ, USA) at 488 nm according to different cell fluorescence intensities at each phrase (G0/G1 phrase, S phrase, and G2/M phrase).

Cell apoptosis was measured by Annexin V-fluorescein isothiocyanate (FITC) and PI double staining. Cells were resuspended in 500 μL Binding buffer and stained by 5 μL Annexin V-FITC staining solution and 10 μL PI solution. Cell apoptosis was also tested by a flow cytometer (BD Bioscience) within 30 min without light exposure. On the scatter plot, living cells in the lower left quadrant (Q4) were FITC^−^/PI^−^, apoptotic cells in the early stage in the lower right quadrant (Q3) were FITC^+^/PI^−^, and necrotic and apoptotic cells in the late stage in the upper right quadrant (Q2) were FITC^+^/PI^+^. Apoptosis rate = early apoptosis percentage (Q3) + late apoptosis percentage (Q2).

### Tumor Xenografts in Nude Mice

Tumor growth was observed by establishing a model of NPC in nude mice. Detached by 0.25% trypsin, SUNE-1 and CNE2 cells at logarithmic phase were configured into single cell suspension at 5 × 10^7^ cells/mL. The cell suspension (0.2 mL) was injected to the right armpit of mice by a microinjector to establish mouse models. Modeled mice were raised in a specific pathogen-free environment. Started from the 4th d, tumor growth was observed and the mice were weighed every 4 days. Nude mice were euthanized on the 20th d after injection and tumors were resected, weighed by an electronic balance and photographed.

### Dual Luciferase Reporter Gene Assay

Dual luciferase reporter gene system was adopted to confirm the binding sites of miR-18a and 3′untranslated region (UTR) of TGFBR3 mRNA. A biological prediction website (http://www.microrna.org/microrna/home.do) was used to analyze the target gene of miR-18a, and discover the existence of the complementary binding site of miR-18a on the 3′UTR of TGFBR3. Dual luciferase reporter gene assay was employed to further verify whether TGFBR3 was directly targeted by miR-18a. A pmirGLO-TGFBR3-wild type (WT) and a pmirG-LO-TGFBR3-mutant type (MUT) of TGFBR3 3′UTR binding site were constructed. TGFBR3-WT or TGFBR3-MUT and miR-18a mimics or mimics NC were co-transfected into SUNE-1 and CNE2 cells by Lipofectamine 2000 (Invitrogen) and incubated for 48 h. A luciferase assay kit (Promega, Madison, WI, USA) was utilized to analyze cells.

### Statistical Analysis

SPSS21.0 statistical software (IBM Corp. Armonk, NY, USA) was used for analysis. Data were expressed as mean ± standard deviation. Differences between two groups were analyzed by *t* test while differences among multiple groups by one-way analysis of variance (ANOVA), followed by Tukey’s post hoc test. A significant difference was considered at *P* < 0.05.

## Results

### Identification of M2 Macrophages

The monocytes enriched by adherent method and monocytes induced by M-CSF were collected from peripheral blood of healthy donors. Immunofluorescence detection of CD68, CD206, and CD163 confirmed that PBMCs induced by M-CSF in vitro turned to macrophages with typical molecular characteristics, which met our requirements (Fig. 1a).

**Fig. 1:** Identification of M2 macrophages. **a**. CD68, CD206, and CD163 were expressed on the surface of macrophages obtained after monocyte induction in vitro. **b** Polarized macrophages by IL-4 were M2 macrophages. **c** CD163 was highly expressed and CD68 was lowly expressed in M2 macrophages polarized by IL-4. **d** CCL22 was highly expressed in M2 macrophages. **e** PPAR-γ was highly expressed in M2 macrophages. **f** miR-18a was highly expressed in M2 macrophages; *P < 0.05; **P < 0.01. Measurement data were expressed as mean ± standard deviation, *N* = 3. Comparisons between two groups was analyzed by *t* test

The obtained macrophages were polarized by IL-4 and observed under a microscope for morphology. It was manifested that macrophages (M0) without IL-4 stimulation were diverse and irregular, showing a round, oval, or spindle shape. Stimulated by IL-4, M2 macrophages became larger and predominantly turned to round shape, which were in conformity to the morphological characteristics of M2 macrophages as previously described [20] (Fig. 1b).

Flow cytometry tested the surface antigens of the adherent cells stimulated by 20 ng/mL IL-4 for 24 h and found that CD68 was expressed at 21.16% while CD163 were at 98.69% of the total number of cells (Fig. 1c), confirming the adherent cells being M2 macrophages. RT-qPCR revealed that with M0 cells by contrast, CCL22 and PPAR-γ (typical polarizing molecules) increased in M2 macrophages (Fig. 1d, e), indicating the successful induction of M2 macrophages.

RT-qPCR also manifested that miR-18a expression increased in M2 macrophages in contrast to the M0 macrophages (*P* ˂ 0.05) (Fig. 1f).

### MiR-18a Is Highly Expressed and TGFBR3 Is Poorly Expressed in NPC Cells

Bioinformatics website (miRanda) predicted the potential targets of miR-18a and TGFBR3 was considered as one target of miR-18a (Fig. 2a). Dual luciferase reporter gene assay was implemented to verify that miR-18a targeted 3′UTR of TGFBR3. TGFBR3-WT or TGFBR3-MUT were cloned into the pmirGLO vector and co-transfected with miR-18a mimics or NC into SUNE-1 and CNE2 cells. miR-18a mimics had no influence on the luciferase activity of TGFBR3 3′UTR-MUT but impaired that of TGFBR3 3′UTR-WT in SUNE-1 and CNE2 cells, suggesting that TGFBR3 was a target gene regulated by miR-18a (Fig. 2b).

**Fig. 2:** MiR-18a is highly expressed and TGFBR3 is poorly expressed in NPC cells. **a** miRanda predicted miR-18a targeting TGFBR3. **b** Dual luciferase reporter gene assay verified miR-18a targeting TGFBR3. **c** miR-18a expression was elevated and TGFBR3 expression was decreased in miR-18a mimics-transfected M2 macrophages. **d** miR-18a expression was decreased and TGFBR3 expression was elevated in miR-18a inhibitors-transfected M2 macrophages. **e** miR-18a expression was elevated and TGFBR3 expression was decreased in NPC cell lines versus to NP96 cells. **f** miR-18a expression was elevated and TGFBR3 expression was decreased in miR-18a mimics-transfected SUNE-1 cells. **g** miR-18a expression was decreased and TGFBR3 expression was elevated in miR-18a inhibitors-transfected CNE2 cells. **h** miR-18a expression was elevated and TGFBR3 expression was decreased in SUNE-1 cells co-cultured with miR-18a mimics-transfected M2 macrophages. **i** miR-18a expression was decreased and TGFBR3 expression was elevated in CNE2 cells co-cultured with miR-18a inhibitors-transfected M2 macrophages; *P < 0.05; **P < 0.01. Measurement data were expressed as mean ± standard deviation, *N* = 3. Comparisons between two groups were analyzed by *t* test. Comparisons among multiple groups were analyzed by one-way ANOVA, followed by Tukey’s post hoc test

The transfection efficiency of miR-18a mimics or miR-18a inhibitors in M2 macrophages was manifested by determination of miR-18a and TGFBR3 expression in M2 macrophages by RT-qPCR and Western blot assay. It was obvious that (Fig. 2c, d) miR-18a overexpression elevated miR-18a expression and reduced TGFBR3 expression in M2 macrophages. Oppositely, miR-18a inhibition reduced miR-18a expression and increased TGFBR expression in M2 macrophages. No difference was witnessed in the miR-18a expression while TGFBR3 expression lessened when M2 macrophages transfected with si-TGFBR3. No difference was witnessed in the miR-18a expression while TGFBR3 expression grew upon OE-TGFBR3 transfection to M2 macrophages.

miR-18a and TGFBR3 expression in CNE2, TW03, C666-1, SUNE-1, and NP96 cell lines were tested by RT-qPCR and Western blot assay. In NPC cells, by comparison with NP96 cells, miR-18a expression increased and TGFBR3 expression decreased (Fig. 2e). Due to CNE2 cells and SUNE-1 cells manifested with the largest and the smallest differences in miR-18a expression from NP96 cells, they were selected for the proceeding miRNA downregulation and upregulation assays, respectively.

To identify the effects of miR-18a and TGFBR3 on NPC cells, SUNE-1 cells were transfected with miR-18a mimics or si-TGFBR3 while CNE2 cells with miR-18a inhibitors or OE-TGFBR3. RT-qPCR and Western blot assay demonstrated that miR-18a mimics elevated miR-18a expression and reduced TGFBR3 expression in SUNE-1 cells. Transfection of si-TGFBR3 had no effect on miR-18a expression while reduced TGFBR3 expression in SUNE-1 cells. miR-18a inhibitors decreased miR-18a expression and elevated TGFBR3 expression in CNE2 cells. OE-TGFBR3 transfection in CNE2 cells did not affect miR-18a expression but elevated TGFBR3 expression (Fig. 2f, g).

To explore the effects of miR-18a from M2 macrophages on NPC cells, miR-18a mimics- or si-TGFBR3-transfected M2 macrophages or miR-18a inhibitors- or OE-TGFBR3-transfected M2 macrophages were co-cultured with SUNE-1 or CNE2 cells in the Transwell chamber, respectively. RT-qPCR and Western blot assay tested miR-18a and TGFBR3 expression in SUNE-1 or CNE2 cells. SUNE-1 cells co-cultured with untransfected or miR-18a mimics-transfected M2 macrophages demonstrated with raised miR-18a expression and degraded TGFBR3 expression. No difference was noticed in the miR-18a expression and TGFBR3 expression reduced in SUNE-1 cells which had co-cultured with si-TGFBR3-transfected M2 macrophages (Fig. 2h). After co-culture with untransfected M2 macrophages, CNE2 cells were featured by increased miR-18a expression and decreased TGFBR3 expression. However, reduced miR-18a expression and elevated TGFBR3 expression presented in CNE2 cells which were in advance co-cultured with miR-18a inhibitors-transfected M2 macrophages. No difference was recognized in the miR-18a expression, and TGFBR3 expression increased in CNE2 cells co-cultured with OE-TGFBR3-transfected M2 macrophages (Fig. 2i).

### miR-18a from M2 Macrophages Promotes NPC Cell Viability and Colony-Forming Ability

MTT assay and colony formation assay were applied to identify the impacts of miR-18a and TGFBR3 on viability and colony-forming ability of SUNE-1 cells and CNE2 cells. miR-18a mimics, miR-18a inhibitors, si-TGFBR3, or OE-TGFBR3 were transfected into SUNE-1 cells or CNE2 cells. It was indicated that in SUNE-1 cells, miR-18a upregulation or TGFBR3 downregulation enhanced cell viability and elevated colony number (Fig. 3a, e). In CNE2 cells, cell viability was impaired and the number of colonies was reduced by miR-18a inhibition or TGFBR3 overexpression (Fig. 3b, f).

**Fig. 3:** miR-18a from M2 macrophages induces NPC cell viability and colony-forming ability. **a** miR-18a mimics or si-TGFBR3 increased viability of SUNE-1 cells. **b** miR-18a inhibitors or OE-TGFBR3 decreased viability of CNE2 cells. **c** Co-culture with miR-18a mimics- or si-TGFBR3-transfected M2 macrophages increased viability of SUNE-1 cells. **d** Co-culture with miR-18a inhibitors or OE-TGFBR3-transfected M2 macrophages decreased viability of CNE2 cells. **e** miR-18a mimics or si-TGFBR3 increased colony number of SUNE-1 cells. **f** miR-18a inhibitors or OE-TGFBR3 decreased colony number of CNE2 cells. **g** Co-culture with miR-18a mimics- or si-TGFBR3-transfected M2 macrophages increased colony number of SUNE-1 cells. **h** Co-culture with miR-18a inhibitors or OE-TGFBR3-transfected M2 macrophages decreased colony number of CNE2 cells; *P < 0.05; **P < 0.01. Measurement data were expressed as mean ± standard deviation, *N* = 3. Comparisons among multiple groups were analyzed by one-way ANOVA, followed by Tukey’s post hoc test

To examine the effects of miR-18a from M2 macrophage on viability and colony formation ability of NPC cells, miR-18a mimics-, miR-18a inhibitors-, si-TGFBR3-, or OE-TGFBR3-transfected M2 macrophages were co-cultured with SUNE-1 cells or CNE2 cells in the Transwell chamber. MTT and colony formation assay displayed that SUNE-1 cells co-cultured with untransfected, or miR-18a mimics-transfected or si-TGFBR3-transfected M2 macrophages were presented with reinforced cell viability and increased number of colonies (Fig. 3c, g).

CNE2 cells co-cultured with untransfected M2 macrophages were highlighted with strengthened cell viability and increased colonies. However, CNE2 cells co-cultured with either miR-18a inhibitors-transfected or OE-TGFBR-transfected M2 macrophages were exhibited with diminished cell viability and decreased colonies (Fig. 3d, h).

### miR-18a from M2 Macrophages Promotes NPC Cell Invasion and Migration Abilities

For better comprehension of how miR-18a and TGFBR3 affected migration and invasion of NPC cells, scratch test and Transwell assay were implemented. The results disclosed that SUNE-1 cells transfected with miR-18a mimics or si-TGFBR3 were characterized by increased cell migration distance and invasion cells (Figs. 4a and 5a).

**Fig. 4:** miR-18a from M2 macrophages promotes NPC cell migration ability. **a** miR-18a mimics or si-TGFBR3 increased migration of SUNE-1 cells. **b** miR-18a inhibitors or OE-TGFBR3 decreased migration of CNE2 cells. **c** Co-culture with miR-18a mimics- or si-TGFBR3-transfected M2 macrophages increased migration of SUNE-1 cells. **d** Co-culture with miR-18a inhibitors or OE-TGFBR3-transfected M2 macrophages decreased migration of CNE2 cells; *P < 0.05; **P < 0.01. Measurement data were expressed as mean ± standard deviation, *N* = 3. Comparisons among multiple groups were analyzed by one-way ANOVA, followed by Tukey’s post hoc test

**Fig. 5:** miR-18a from M2 macrophages promotes NPC cell invasion ability. **a** miR-18a mimics or si-TGFBR3 increased invasion of SUNE-1 cells. **b** miR-18a inhibitors or OE-TGFBR3 decreased invasion of CNE2 cells. **c** Co-culture with miR-18a mimics- or si-TGFBR3-transfected M2 macrophages increased invasion of SUNE-1 cells. **b** Co-culture with miR-18a inhibitors or OE-TGFBR3-transfected M2 macrophages decreased invasion of CNE2 cells; *P < 0.05; **P < 0.01. Measurement data were expressed as mean ± standard deviation, *N* = 3. Comparisons among multiple groups were analyzed by one-way ANOVA, followed by Tukey’s post hoc test

In CNE2 cells transfected with miR-18a inhibitors or OE-TGFBR3, the reductions appeared in cell migration distance and invasion cells (Figs. 4b and 5b).

How miR-18a from M2 macrophages influenced invasion and migration abilities of NPC cells were deciphered by miR-18a mimics-, miR-18a inhibitors-, si-TGFBR3-, or OE-TGFBR3-transfected M2 macrophages co-culturing with SUNE-1 or CNE2 cells. The results highlighted that SUNE-1 cells co-cultured with untransfected, or miR-18a mimics-transfected or si-TGFBR3-transfected M2 macrophages were manifested with increased cell migration distance and invasion cells (Figs. 4c and 5c).

Both cell migration distance and invasion cells increased in CNE2 cells co-cultured with untransfected M2 macrophages. Upon co-culture with miR-18a inhibitors-transfected or OE-TGFBR3-transfected M2 macrophages, CNE2 cells were showed with reduced migration distance and invasion cells (Figs. 4d and 5d).

### miR-18a from M2 Macrophages Arrests Fewer NPC Cell at G0/G1 Phase and Suppresses Apoptosis

Cell cycle distribution and apoptosis were tested by flow cytometry to stratify the effects of miR-18a and TGFBR3 on NPC cells. It was indicated that transfection of miR-18a mimics or si-TGFBR3 reduced SUNE-1 cells arrested in the G0/G1 phase, increased cells in the S and G2/M phases, and reduced cell apoptosis rate (Figs. 6a and 7a).

**Fig. 6:** miR-18a from M2 macrophages arrests fewer NPC cell at G0/G1 phase. **a** miR-18a mimics or si-TGFBR3 decreased SUNE-1 cells in the G0/G1 phase, and increased SUNE-1 cells in the S and G2/M phases. **b** miR-18a inhibitors or OE-TGFBR3 increased CNE2 cells in the G0/G1 phase, and decreased CNE2 cells in the S and G2/M phases. **c** Co-culture with miR-18a mimics- or si-TGFBR3-transfected M2 macrophages decreased SUNE-1 cells in the G0/G1 phase, and increased SUNE-1 cells in the S and G2/M phases. **d** Co-culture with miR-18a inhibitors or OE-TGFBR3-transfected M2 macrophages increased CNE2 cells in the G0/G1 phase, and decreased CNE2 cells in the S and G2/M phases; *P < 0.05; **P < 0.01. Measurement data were expressed as mean ± standard deviation, *N* = 3. Comparisons among multiple groups were analyzed by one-way ANOVA, followed by Tukey’s post hoc test

**Fig. 7:** miR-18a from M2 macrophages inhibits NPC cell apoptosis. **a** miR-18a mimics or si-TGFBR3 decreased apoptosis of SUNE-1 cells. **b** miR-18a inhibitors or OE-TGFBR3 increased apoptosis of CNE2 cells. **c** Co-culture with miR-18a mimics- or si-TGFBR3-transfected M2 macrophages decreased apoptosis of SUNE-1 cells. **d** Co-culture with miR-18a inhibitors or OE-TGFBR3-transfected M2 macrophages increased apoptosis of CNE2 cells; *P < 0.05; **P < 0.01. Measurement data were expressed as mean ± standard deviation, *N* = 3. Comparisons among multiple groups were analyzed by one-way ANOVA, followed by Tukey’s post hoc test

Upon transfection with miR-18a inhibitors or OE-TGFBR3, CNE2 cells in the G0/G1 phase trended toward an elevation while those in the S and G2/M phases toward a reduction, and cell apoptosis rate raised (Figs. 6b and 7b).

With the purpose to decode the mechanism of miR-18a from M2 macrophages in NPC cell cycle distribution and apoptosis, M2 macrophages transfected with miR-18a mimics, miR-18a inhibitors, si-TGFBR3, or OE-TGFBR3 were co-cultured with SUNE-1 cells or CNE2 cells in the Transwell chamber. Co-cultured with untransfected, or miR-18a mimics-transfected or si-TGFBR3-transfected M2 macrophages, reduced SUNE-1 cells were displayed in the G0/G1 phase and increased cells in the S and G2/M phases, and SUNE-1 cell apoptosis rate decreased (Figs. 6c and 7c).

Co-cultured with untransfected M2 macrophages, CNE2 cells in the G0/G1 phase reduced, cells in the S and G2/M phases increased, and apoptosis rate declined. On the contrary, co-cultured with miR-18a inhibitors-transfected or OE-TGFBR3-transfected M2 macrophages, CNE2 cells in the G0/G1 phase elevated while those in the S and G2/M phases decreased, and apoptosis rate elevated (Figs. 6d and 7d).

### miR-18a from M2 Macrophages Reduces p-Smad1/t-Smad1 and Elevates p-Smad3/t-Smad3 in NPC Cells

Western blot assay detected TGF signaling pathway-related proteins in NPC cells to further explain the effects of miR-18a and TGFBR3 on TGF signaling pathway.

It was explained that transfection of miR-18a mimics or si-TGFBR3 reduced p-Smad1/t-Smad1 and elevated p-Smad3/t-Smad3 in SUNE-1 cells (Fig. 8a).

**Fig. 8:** miR-18a from M2 macrophages decreases p-Smad1/t-Smad1 and increases p-Smad3/t-Smad3 in NPC cells. **a** miR-18a mimics or si-TGFBR3 in SUNE-1 cells decreased p-Smad1/t-Smad1 and elevated p-Smad3/t-Smad3. **b** miR-18a inhibitors or OE-TGFBR3 in CNE2 cells increased p-Smad1/t-Smad1 and decreased p-Smad3/t-Smad3. **c** Co-culture with miR-18a mimics- or si-TGFBR3-transfected M2 macrophages decreased p-Smad1/t-Smad1 and elevated p-Smad3/t-Smad3. **d** Co-culture with miR-18a inhibitors or OE-TGFBR3-transfected M2 macrophages increased p-Smad1/t-Smad1 and decreased p-Smad3/t-Smad3; *P < 0.05; **P < 0.01. Measurement data were expressed as mean ± standard deviation, *N* = 3. Comparisons among multiple groups were analyzed by one-way ANOVA, followed by Tukey’s post hoc test

Transfection with miR-18a inhibitors or OE-TGFBR3 led to declined p-Smad3/t-Smad3 and increased p-Smad1/t-Smad1 in CNE2 cells (Fig. 8b).

miR-18a from M2 macrophages influencing TGF signaling pathway in NPC cells was determined by Western blot assay through testing TGF signaling pathway-related proteins in SUNE-1 cells and CNE2 cells which had co-cultured with miR-18a mimics-, miR-18a inhibitors-, si-TGFBR3-, or OE-TGFBR3-transfected M2 macrophages in the Transwell chamber.

SUNE-1 cells co-cultured with untransfected, miR-18a mimics-transfected, or si-TGFBR3-transfected M2 macrophages were manifested with reduced p-Smad1/t-Smad1 and incremental p-Smad3/t-Smad3 (Fig. 8c).

Co-cultured with untransfected M2 macrophages, CNE2 cells trended toward declined p-Smad1/t-Smad1 and elevated p-Smad3/t-Smad3. In an opposite way, CNE2 cells were demonstrated with increased p-Smad1/t-Smad1 and decreased p-Smad3/t-Smad3 when co-cultured with miR-18a inhibitors-transfected or OE-TGFBR3-transfected M2 macrophages (Fig. 8d).

### miR-18a from M2 Macrophages Induces Tumor Growth in Nude Mice with NPC

Tumor xenografts were conducted on nude mice to further elucidate the impacts of miR-18a and TGFBR3 on tumor growth of NPC.

It was indicated that injected with miR-18a mimics-transfected or si-TGFBR3-transfected SUNE-1 cells, mice were manifested with enlarged tumor volume and heavier tumor weight (Fig. 9a).

**Fig. 9:** miR-18a from M2 macrophages promotes tumor growth in nude mice with NPC. **a** miR-18a mimics or si-TGFBR3 in SUNE-1 cells increased tumor volume and weight. **b** miR-18a inhibitors or OE-TGFBR3 in CNE2 cells decreased tumor volume and weight. **c** Co-culture with miR-18a mimics- or si-TGFBR3-transfected M2 macrophages increased tumor volume and weight. **d** Co-culture with miR-18a inhibitors or OE-TGFBR3-transfected M2 macrophages decreased tumor volume and weight; *P < 0.05; **P < 0.01. Measurement data were expressed as mean ± standard deviation, three nude mice in each group. Comparisons among multiple groups were analyzed by one-way ANOVA, followed by Tukey’s post hoc test

Reduced tumor volume and weight were presented in mice with injection of miR-18a inhibitors-transfected or OE-TGFBR3-transfected CNE2 cells (Fig. 9b).

Tumor growth was observed in mice which had injected with miR-18a mimics-, miR-18a inhibitors-, si-TGFBR3-, or OE-TGFBR3-transfected M2 macrophages to illustrate the mechanism of miR-18a from M2 macrophages in NPC.

After co-culture with untransfected, miR-18a mimics-transfected or si-TGFBR3-transfected M2 macrophages, SUNE-1 cells were injected into mice and mice were observed with larger tumor volume and heavier tumor weight (Fig. 9c).

CNE2 cells were co-cultured with M2 macrophages and injected into mice with the results suggesting growing tumor volume and weight. Both tumor volume and weight were inclined to reduce when mice were injected with CNE2 cells which had co-cultured with miR-18a inhibitors-transfected or OE-TGFBR3-transfected M2 macrophages (Fig. 9d).

## Discussion

NPC refers to a polygenic disease threatened by a wide range of factors [21]. MiRNAs are previously implied to participate in the pathogenesis of NPC via regulation of their target genes which are indicators of cellular processes and pathways [22]. Concretely, miR-18a advances NPC progression by miRNA biogenesis impairing [6]. Given that this study goes forward to decipher the combined interactions of miR-18a from M2 macrophages and TGFBR3 in NPC with the conclusion elucidating that miR-18a from M2 macrophages stimulates NPC progression via TGFBR3 inhibition (Fig. 10).

**Fig. 10:** Schematic representation of macrophage-derived exosomal miR-18a in NPC and the involvement of TGFBR3-mediated TGF-β signaling pathway

At the start of this study, macrophages are stimulated by IL-4 to differentiate to M2 macrophages which are found to enrich the expression of miR-18a. As we know, during macrophage polarization, miRNA’s expression was altered [23]. In addition, M2 polarization enriches genes which are involved in the cell cycle and metabolic processes, and the M2 phenotype is conducive to tumor growth and angiogenesis in neoplastic tissues [24]. Based on the M2 macrophages-enriched miR-18a, a series of experiments were successfully conducted.

Initially, our study has uncovered that miR-18a is highly expressed while TGFBR3 is poorly expressed in NPC cells. Drawn from a previous study, it is concluded that miR-18a is overexpressed in NPC tissues with its association with lymph node metastasis and clinical stage [5]. Besides that, miR-17-92 cluster members including miR-18a are documented to be overexpressed in NPC tissues [25]. Furthermore, upregulated miR-18a is reported to demonstrate in NPC tissues which is connected with tumor node metastasis stage and tumor size [4]. Experimentally, except for the downregulated TGFBR3 in tongue squamous cell carcinoma [26], there has been another study depicting reduced TGFBR3 in clear-cell renal cell carcinomas accompanied by unwanted prognosis [27]. Anyhow, the results in this study are consistent with these study findings to some extent.

In order to explore the roles of miR-18a and TGFBR3 in NPC cell progression, we have conducted a series of assays with the results indicating that upregulated miR-18a or downregulated TGFBR3 triggers NPC cell progression while miR-18a repression or TGFBR3 elevation has the opposite effects on NPC cells. Widely, suppression of miR-18a is evidenced to hamper cell progression in malignancies including ovarian cancer, colitis-associated colorectal cancer, and hepatocellular carcinoma [28–30]. Narrowly, an existed study has pronounced that upregulated miR-18a promotes NPC cell progression via mediation of DICER1 [6]. In addition, it is noticed that overexpressed miR-18a in NPC is believed to connect with NPC metastasis and repressed miR-18a partially contributes to better prognosis of NPC patients [31]. Lately, it is surveyed that downregulation of miR-18a is capable of discouraging NPC proliferation, invasion, and migration [4]. Additionally, a decrease in TGFBR3 expression is regarded to link with laryngeal squamous cell carcinoma (LSCC) invasion and miR-223/TGFBR3 axis regulation takes part in LSCC progression inhibition [32]. TGFBR3 elevation is documented to restrict NPC cell viability, induce apoptosis, and activate pro-apoptosis signaling pathways [14]. Previously, a study has indicated that upregulation of TGFBR3 promotes apoptosis and cells arrested in the G2/M phase, resulting in impaired cell viability and migration in salivary gland adenoid cystic carcinoma [33]. Intriguingly, it is formerly described that induction of TGFBR3 contributes to disrupt intrahepatic cholangiocarcinoma progression [34].

Despite the protective role of lowly expressed miR-18a and overexpressed TGFBR3 in NPC cell in vitro, we have performed tumor xenografts in nude mince in vivo for further verification with the results explaining that miR-18a knockdown or TGFBR3 elevation restrains tumor growth in nude mice. As demonstrated in a prior study, miR-18a-injected nude mice show with enhanced tumor growth [5] and conversely, the miR-18a antagomir-injected nude mice are displayed with suppressed tumor growth in NPC [4]. In the light of the TGFBR3 reduction in tumor growth, it is suggested that poorly expressed TGFBR3 provokes tumor formation in clear-cell renal cell carcinoma [27]. In the opposite way, an increase in TGFBR3 is recognized to hinder tumor growth in lung cancer with the presence of long non-coding RNA ADAM metallopeptidase with thrombospondin type 1 motif, 9 antisense RNA 2 elevation, and miR-223-3p suppression [35]. This study has also predicted and verified that TGFBR3 is a target gene of miR-18a. But, more studies still need to be conducted for further verification.

## Conclusion

Generally speaking, this study elaborates the concrete mechanisms that miR-18a from M2 macrophages inhibits TGFBR3 expression to exacerbate the progression of NPC via TGF-β signaling pathway, the results of which is abrogated by miR-18a knockdown or TGFBR3 elevation. This study updates the therapeutic target for NPC. However, a large cohort researches are still in need for in-depth explorations.

## Data Availability

Not applicable.
